# Advancements in stem cell-derived hepatocyte-like cell models for hepatotoxicity testing

**DOI:** 10.1186/s13287-021-02152-9

**Published:** 2021-01-25

**Authors:** Meixian Jin, Xiao Yi, Wei Liao, Qi Chen, Wanren Yang, Yang Li, Shao Li, Yi Gao, Qing Peng, Shuqin Zhou

**Affiliations:** 1 Department of Anesthesiology, Zhujiang Hospital, Southern Medical University, Guangzhou, 510000 China; 2 Department of Gynecology, Zhujiang Hospital, Southern Medical University, Guangzhou, China; 3 General Surgery Center, Department of Hepatobiliary Surgery II, Guangdong Provincial Research Center for Artificial Organ and Tissue Engineering, Guangzhou Clinical Research and Transformation Center for Artificial Liver, Institute of Regenerative Medicine, Zhujiang Hospital, Southern Medical University, Guangzhou, Guangdong Province China

**Keywords:** Stem cells, Hepatocyte-like cells, Drug screening, Drug-induced liver injury, 3D cell culture

## Abstract

Drug-induced liver injury (DILI) is one of the leading causes of clinical trial failures and high drug attrition rates. Currently, the commonly used hepatocyte models include primary human hepatocytes (PHHs), animal models, and hepatic cell lines. However, these models have disadvantages that include species-specific differences or inconvenient cell extraction methods. Therefore, a novel, inexpensive, efficient, and accurate model that can be applied to drug screening is urgently needed. Owing to their self-renewable ability, source abundance, and multipotent competence, stem cells are stable sources of drug hepatotoxicity screening models. Because 3D culture can mimic the in vivo microenvironment more accurately than can 2D culture, the former is commonly used for hepatocyte culture and drug screening. In this review, we introduce the different sources of stem cells used to generate hepatocyte-like cells and the models for hepatotoxicity testing that use stem cell-derived hepatocyte-like cells.

## Introduction

Drug-induced liver injury (DILI) is one of the main reasons for the withdrawal of new drugs from the market and is also an important factor leading to the failure of drug development. In Western countries, the annual incidence of DILI is 1 to 20 cases per 100,000 inhabitants [1–3]. In China, a retrospective study found an estimated incidence of 23.8 DILI cases per 100,000 persons per year, which is higher than that reported for Western countries [4]. The safety of drugs has always been a focus, and finding a reasonable and efficient drug prediction model is a great challenge in the pharmaceutical field [5].

DILI can be divided into intrinsic or idiosyncratic DILI (iDILI). Intrinsic DILI is typically dose-related and predictable. It transpires within a short period and shows insignificant individual differences. iDILI is less commonly seen in clinical practice; it is unpredictable and features significant individual differences related to age, sex, genetic factors, the environment, and associated basic diseases. Thus, the assessment of iDILI is one of the most challenging liver diseases for hepatologists because of its relatively low incidence, distinct individual differences, diverse manifestations, and lack of typical biomarkers [6–8].

Various hepatocyte models have been developed for drug safety tests (Table 1).

**Table 1:** Advantages and disadvantages of using human hepatocytes or stem cell-derived hepatocyte-like cells for drug screening

Cell types	Descriptions	Advantages	Disadvantages	References
Primary human hepatocytes	Hepatocytes isolated from fresh human liver	Maintain original structure and functions, the gold standard	Limited availability, rapid dedifferentiation, and function loss	[9, 10]
Hepatic cell lines	Immortalized cell lines from human liver carcinoma cells, e.g., HepG2, Hep3B and Huh7	Easy obtainment and low cost	Loss of original characteristics of hepatocytes and inaccurate predictions	[11]
hESCs-derived HLCs	Hepatocytes differentiated from hESCs by mimicking the developmental pathway of the liver during embryogenesis	High self-renewal and pluripotency	Ethical issues	[12]
hiPSCs-derived HLCs	Hepatocytes differentiated from hiPSCs that are obtained by reprogramming of adult somatic cells	Self-renewal and pluripotency, no ethical issues, and potential to model iDILI	Low reprogramming efficiency and potential tumorigenic risk	[13, 14]
hMSCs-derived HLCs	Hepatocytes differentiated from hMSCs that can be obtained from adipose tissue, bone marrow, placenta, etc.	Abundant sources, fewer ethical concerns, and lower tumorigenic risk	Relatively low endoderm differentiation potential	[15, 16]
Transdifferentiated cells	Hepatocytes transdifferentiated directly from human adult somatic cells	Fewer operational steps	Low reprogramming efficiency, limited proliferation capacity	[17, 18]
HepaRG cells	A human bipotent progenitor cell line that can be differentiated into hepatocytes	High levels of major phase I and phase II enzymes	Low functional levels of CYP2D6, CYP2A6, and CYP2E1	[19–21]

*hESCs* human embryonic stem cells, *HLCs* hepatocyte-like cells, *hiPSCs* human induced pluripotent stem cells, *hMSCs* human mesenchymal stem cells, *iDILI* idiosyncratic drug-induced liver injury, *CYP* cytochrome P450

With considerable interspecies differences in drug metabolism, animal models cannot accurately reflect the metabolic response of drugs in humans, and high costs and ethical issues also limit the application of animal models [22]. Isolated primary human hepatocytes (PHHs) maintain their original structure and most of their function in vivo, so they are an ideal model for evaluating drug metabolism and toxicity and thus are “gold standard” models for drug testing [9]. However, their rapid phenotype change and short life span seriously affect the accuracy of predicting drug metabolism [10, 23]. Hepatic cell lines are inexpensive and can reproduce indefinitely, but they lose the original characteristics of hepatocytes in long-term culture in vitro and cannot effectively reflect the complex metabolic effects of drugs in vivo [11].

Recently, stem cells have been widely used in regenerative medicine, safety pharmacology, toxicology research, regenerative medicine, and cell therapy. Because of their source abundance, self-renewable ability, high proliferative potential, and multipotent competences, stem cells are stable sources of hepatocytes for safe pharmacology and toxicology evaluation. In this sense, stem cell-derived hepatocytes are able to overcome the shortcomings of traditional hepatocyte models, such as interspecies differences and insufficient cellular function. Three-dimensional (3D) culture technology has enabled the formation of cell–cell and cell–matrix interactions and can better maintain cell activity and function; hence, with 3D culture, liver tissue engineering has undergone a paradigm shift from classic monolayer cell culture to more advanced organotypic liver models [24]. With the rapid development of stem cell technology, scientists are paying more attention to stem cells, hoping to establish a more effective evaluation model of hepatotoxicity in vitro by using stem cells [25]. In addition, the use of stem cells allows for assessing drug toxicity in vivo. Also, humanized mouse models based on stem cell-derived hepatocytes provide good information about drug metabolism, disposition, and toxicity in humans and can contribute to the development of personalized medicine strategies, which would improve drug efficacy and safety [26]. Studies of “hepatocytes” derived from stem cells have focused on generating a closer representation of the mature PHH phenotype, and the term hepatocyte-like cells (HLCs) is commonly used to describe these cells [27].

In this review, we focus on the technology of stem cell differentiation into HLCs and the current uses of stem cells for hepatotoxicity evaluation.

## Generation of hepatocyte-like cells from stem cells

### hESCs, hiPSCs, and hMSCs

Thomson et al. [12] found that the human embryonic stem cells (hESCs) expressed high levels of telomerase activity, so these cells still maintained the developmental potential to form trophoblast and derivatives of all three embryonic germ layers even after undifferentiated proliferation in vitro for a long time. Although hESCs have high self-renewing potency and pluripotency, their use is limited owing to the ethical issues involved in the process of separation. Induced pluripotent stem cells are reprogrammed from adult somatic cells by introducing four factors: Oct3/4, Sox2, c-Myc, and Klf4. These cells exhibit a gene expression pattern, epigenetic profile, and differentiation potential similar to hESCs [28]. Because they are easy to obtain without evoking ethical problems and have unique advantages in the study of iDILI, the use of human induced pluripotent stem cells (hiPSCs) differentiated into hepatocytes has gradually become a research hotspot [13, 14]. Human mesenchymal stem cells (hMSCs) can be isolated from various somatic tissues, such as adipose tissue, bone marrow, placenta, umbilical cord, and menstrual blood [15, 29–32]. As compared with hESCs/hiPSCs, the use of hMSCs leads to fewer ethical concerns, and the tumorigenesis risk is also lower, but the expansion capacity and ability to differentiate into endoderm are relatively lower [16].

Most of the current protocols attempt to promote the differentiation of stem cells by mimicking the development of the liver during embryogenesis in three steps: definitive endoderm differentiation, hepatocyte differentiation, and hepatocyte maturation. Hepatic growth factor, fibroblast growth factor, activin A, oncostatin M, and other cytokines play important roles in different differentiation stages [33–36]. In the current methods, HLCs exhibit an immature hepatic phenotype (e.g., express fetal markers such as alpha fetoprotein) [37, 38]. In particular, the gene expression and enzyme activity of cytochromes P450 (CYPs) are far less than those of PHHs in hiPSC-derived HLCs [39, 40]. Another study showed that as compared with PHHs, many genes in HLCs involved in xenobiotic metabolism remain low, and gene regulatory network analysis showed that HLCs contain features of not only liver but also stem cells, intestine, and fibroblasts [41]. Therefore, the induction protocol needs to be further optimized before using HLCs as an alternative to hepatocytes in drug research.

Researchers have shown that the use of small molecules [42, 43] regulating the extracellular nutrient level [44, 45], inducing overexpression of hepatic transcription factors [46, 47], and manipulating miRNA expression [48, 49] represents powerful methods for the efficient generation of metabolically functional hepatocytes. However, substantial variation in differentiation efficiencies has been observed among different stem cell lines, and a set of consensus criteria is needed to assess whether HLCs are suitable for drug testing. In this regard, some experts suggest that drug screening systems should be evaluated in terms of the viability, morphology, functionality, and toxicity features [50].

### Transdifferentiation

Researchers have tried to skip over iPSC differentiation and directly convert terminally differentiated cells into hepatocytes [51]. Huang et al. demonstrated that overexpression of transcription factors such as FOXA3, HNF1A, and HNF4A directly induced fibroblasts into human-induced hepatocytes (hiHeps). Although hiHeps express hepatic gene programs and display functions characteristic of hepatocytes, there is still a large gap in cell metabolic rate between hiHeps and primary hepatocytes [17]. In addition, Fu et al. [18] described a protocol for achieving the efficient conversion of human primary hepatocytes into liver progenitor-like cells by the delivery of developmentally relevant cues, including NAD+-dependent deacetylase SIRT1 signaling. These progenitor-like cells can re-differentiate to achieve mature hepatic functions. However, the cells feature individual variation: most cannot be cultured beyond 20 passages, and they show reduced proliferation capacity, reduced expression of progenitor markers, and chromosomal abnormalities in the late passage.

### HepaRG cells

The HepaRG cell line is a human bipotent progenitor cell line that can be differentiated into HLCs and biliary epithelial cells [19]. Whole-genome expression profiling showed that HepaRG cells are remarkably similar to human hepatocyte populations [52]. In fact, HepaRG cells maintain liver cell functions, drug-metabolizing enzymes, hepatobiliary transporters, and nuclear receptors better than do other hepatic cell lines [53]. A multiparametric screening assay showed that oxidative stress, mitochondrial damage, and disorders of neutral lipid metabolism were changed notably in HepaRG cells exposed to DILI-related drugs, which accounts for their high sensitivity as compared with other cell lines [54]. A high concentration of DMSO required in standard differentiation protocols limits the use of HepaRG cells [55, 56], but studies have shown that 3D culture or a cocktail of soluble molecules can be used as an alternative to the DMSO-based differentiation protocol for HepaRG [57, 58]. In addition, even though HepaRG cells express high functional levels of most phase I and II enzymes, the levels of some metabolic enzymes such as cytochromes P450 2A6 (CYP2A6), CYP2D6, and CYP2E1 still remain low [20, 21].

## Hepatocyte-like cell models for hepatotoxicity testing

### 2D models

2D monolayer cell culture is a traditional in vitro model for studying the response of cells to drugs that has the advantages of easy and low-cost operation. A few studies have applied stem cell-derived hepatocytes for drug toxicity testing, demonstrating their sensitivity and predictive power in identifying drugs with hepatoxic effects. Although the hepatocyte-like cell model is not as good as that of primary hepatocytes in some respects, the accuracy of drug prediction is far higher than that of hepatic cell lines [59, 60]. An analysis of 12 compounds showed an R2 correlation coefficient of 0.94 for TC50 values obtained for stem cell-derived hepatocytes and primary hepatocytes, which was higher than the R2 coefficient of 0.62 obtained for HepG2 cells. Also, HLCs demonstrated all toxicological endpoints typically examined, including steatosis, apoptosis, and cholestasis [61]. In addition to the direct toxic effects of drugs on liver cells, immune reaction is also involved in the pathogenesis of DILI. Proinflammatory and anti-inflammatory cytokine levels are increased when hESC-derived HLCs are treated with acetaminophen or thiazolidinedione. Kim et al. [62] demonstrated the potential of hESC-derived HLCs in an in vitro model system for assessing drug-induced hepatotoxic immunological events (Table 2).

**Table 2:** Different hepatocyte-like cell models for hepatotoxicity testing

Models	Descriptions	Advantages	Disadvantages	Applications	References
2D monolayer cell culture	Cells adhere to a solid and flat surface	Easy and low-cost operation	Poor cell–cell and cell–matrix interactions, far different from the environment in vivo, limited enzyme activity	Evaluation of drug metabolism and toxicity, drug–drug interactions, high-throughput drug screening, long-term drug toxicity assessment	[62–64, 67–69]
Complex organoids	Organoids with multiple cell types	Presence of non-parenchymal cells, rich and complex structure	Poor homogeneity and controllability	Specific disease models	[75, 76, 78]
Simplified organoids	Organoids with single-cell type	Good homogeneity and controllability	Relatively simple structure and function	Large-scale drug screening	[82–84]
Scaffold-based organoids	Organoids grown in supportive scaffold	Efficient differentiation, intact vasculature, controllable size, shape, permeability, and porosity	Undefined components, lower stability and repeatability, problems of biocompatibility and cytotoxicity, absorption of test compound by scaffold	Studies of drug metabolism, disease modeling, and implantation in vivo	[86–92, 94, 95]
Scaffold-free organoids	Cells self-aggregate to form organoids	Simple operation, low-cost, high throughput, no compatibility issues, cell–cell and cell–matrix interaction, nutrition, oxygen gradient formation	Hypoxia and necrosis in the center of the organoids	Large-scale drug screening	[97, 99]
Patient-derived organoids	Organoids with patient-specific cells	Donor-specific CYP metabolism and drug responses	Relatively complex operation	Disease modeling, mechanism research, targeted drug screening	[100–105]
Organ-on-a-chip	Organ biomimetic system with organoids grown in a microfluidic chip	Precise and dynamic control of the cellular microenvironment	High-cost, complex operation, need of sophisticated equipment	Prediction of drug absorption, metabolism, and clearance	[108, 118–121]
Chimeric mice with humanized livers	Mouse liver cells are replaced by human hepatocytes	Possessing human drug metabolism and transformation functions, good human relevance	High-cost, time-consuming operation, varying degree of humanization, immune-compromised	Preclinical drug evaluation	[128–130, 136–139]

Furthermore, the HLC model allows for high-throughput drug screening and long-term drug toxicity assessment. Ware et al. [63] used a set of 47 drugs to assess the sensitivity and specificity of iPSC-derived HLCs for DILI predictions based on a micropatterned co-culture system. For 37 of these hepatotoxic drugs, the sensitivity of the HLCs and PHHs was 65% and 70%, respectively, with a specificity of 100% for the 10 non-hepatotoxic drugs. Thus, HLCs were quite sensitive and specific to the detection of drug toxicity as compared with PHHs. Long-term culture of HLCs is needed for evaluating chronic hepatoxicity. Holmgren et al. [64] demonstrated that HLCs showed a time-dependent toxic response to amiodarone, aflatoxin B1, and troglitazone when exposed to hepatotoxic compounds for 14 days. Unfortunately, the study lacked data on primary hepatocytes and compared HLCs with only HepG2 cells.

### 3D organoid models

Cells are exposed to a dynamic environment in vivo. The oxygen gradient, nutrient concentration, fluid shear stress, and fluid friction force may significantly affect the hepatic differentiation of stem cells [65, 66]. The static monolayer 2D culture model does not reproduce these conditions, so it cannot maintain the complete drug metabolic capacity of the cells, which may result in non-predictive or misleading data for in vivo drug responses. However, a 3D culture is able to mimic in vivo nutrient and oxygen concentration gradient as well as cell–cell and cell–matrix interactions, has greater stability, and promotes a longer lifespan than does 2D cell culture. Whether stem cells are differentiated or used for predicting drug toxicity, a 3D system is better than a 2D system [67–69]. In recent years, 3D culture technology has developed rapidly and is now used for the development of organoids, spheroids, scaffolds, bioreactors, microfluidic devices, and 3D bioprinting. Organoid technology is one of the most promising 3D models for various applications in regenerative medicine, disease modeling, drug discovery, and hepatotoxicity [70] (Table 2).

Organoids create structures that resemble their organ of origin by assembling themselves into a 3D structure while growing and expanding in vitro. Because organoid models can reproduce organ-specific characteristics, including cellular architecture, morphology, and function, organoid technology has emerged as a powerful and revolutionary strategy enabling studies of disease and has applications for drug discovery and clinical treatments (Fig. 1). However, in the last decade, the meaning of “organoid” has come to encompass a range of cell culture techniques, not necessarily a single technique [71]. Here, we define an organoid as an in vitro 3D cellular cluster derived exclusively from primary tissue, pluripotent stem cells or progenitor cells that is capable of self-renewal and self-organization and exhibits similar organ functionality as the tissue of origin [72–74].

**Fig. 1:** Generation of liver organoid models and their applications. Organoids are formed by a single cell type or with non-parenchymal cells (e.g., endothelial cells) in co-cultures. They can be scaffold-based or scaffold-free. Patient-derived organoids can be applied to disease modeling. Combined with microfluidics, the organ-on-a-chip accurately mimics the microenvironment in vivo. In addition, chimeric mice with humanized livers were introduced for preclinical drug evaluation to further verify drug metabolism and toxicity in vivo. These 3D organoid models can be applied to drug development and drug screening, toxicology mechanism research, regenerative medicine, and personalized therapy

#### Complex and simplified organoids

The liver is mainly composed of hepatocytes, a type of parenchymal cell, but non-parenchymal cells, such as endothelial cells of the hepatic sinus, Kupffer cells, stellate cells, and lymphocytes, also play important roles. Non-parenchymal cells can enhance the maturation of hepatocytes by regulating some key pathways [75, 76]. The ability of human endothelial cells (hECs) to secrete endogenous angiogenic factors might facilitate the recruitment of new blood vessels to the transplantation site [77]; thus, multicellular co-culture is widely used in organoid culture (Fig. 1). HLCs derived from hiPSCs were co-cultured with stromal cell populations, human umbilical vein endothelial cells, and hMSCs on Matrigel matrix to form a vascularized and functional liver tissue mass termed a liver bud. Immunostaining and gene expression analyses revealed a resemblance between in vitro-grown iPSC-derived liver buds and in vivo liver buds [78]. Recently, a variety of different organoid culture methods have been described, and hESCs, hiPSCs, hMSCs, and other stem cells have been reported to form organoids [79–81].

Multicellular co-cultured organoids have abundant structural levels, mimicking the complex niche components and interactions in vivo to a greater extent. However, for drug screening, some experts consider that the organoids should have high prediction power by recapitulating critical aspects of the target in vivo, and simplified procedures are necessary to maintain the homogeneity of the system. Wu et al. [82] established a system to generate hiPSC-derived functional hepato-biliary organoids in vitro without using exogenous cells or DNA transfection. Specifically, this kind of organoid displayed not only hepatocyte function but also the ability to efflux rhodamine and store bile acid. Moreover, after transplantation into immune-deficient mice, the organoids survived for more than 8 weeks. Mun et al. [83] reported that their organoids preserved mature liver properties, including serum protein production, drug metabolism and detoxification functions, active mitochondrial bioenergetics, and regenerative and inflammatory responses. When used for drug screening, the organoids exhibited significant toxic responses to clinically relevant concentrations of drugs that had been withdrawn from the market due to hepatotoxicity. One of the major challenges with the use of hepatic cells in drug screening assays is their loss of detoxification capacity during prolonged cultivation. However, Rashidi et al. [84] reported that their organoids, formed with hiPSCs, exhibited stable CYP3A activity for more than 1 year in culture, thus providing an attractive resource for long-term drug testing in vitro. Moreover, the levels of CYP3A4 and CYP1A2 in the organoids were much higher than those in 2D cultures, and the highest sensitivity to acetaminophen was detected in the organoids even at low concentrations [85].

Thus, for specific disease models, multiplexed organoids accurately mimic the in vivo environment, but simplified organoids with good homogeneity and controllability are more applicable in large-scale drug screening. Both simple and complex culture systems have their pros and cons. How to achieve a balance among efficiency, simplicity, complexity, and controllability needs more exploration.

#### Scaffold-based and scaffold-free organoids

Scaffolds for cell culture are mainly divided into biological and artificial scaffolds. Biocompatibility is better with biological than artificial scaffolds, and the former can better mimic the environment in vivo. Synthetic scaffolds can be used to artificially regulate some characteristics, such as size, shape, hardness, permeability, and porosity, and have better reproducibility and stability than biological scaffolds [86, 87]. Biological scaffolds that are commonly used include natural polymers such as Matrigel, collagen, chitosan, gelatin, cellulose, and alginate. In general, organoid derivation protocols rely mainly on the use of Matrigel. Although Matrigel improves cell growth and efficient differentiation, its complex, ill-defined, and variable components and batch-to-batch variability have led to an uncontrolled cellular microenvironment and reduced repeatability [88]. The use of a natural extracellular matrix (ECM) with better biocompatibility or artificial scaffolds with controlled mechanical characteristics can further define the self-organization of organoids and their functional level. Hydrogels with high biocompatibility and tunable properties, such as permeability, elasticity, stiffness, and chemical reactivity, can mimic the native ECM microenvironment by maintaining spatiotemporal control over biochemical and physical cues [89]. Several defined hydrogels have been shown to facilitate organoid formation as substitutes for Matrigel to improve the reproducibility and maturity of organoids by precisely controlling their componential, structure, and mechanical conditions [90, 91]. In addition, decellularized liver scaffolds provide a biomimetic natural organ scaffold with highly intact native ECM, vascular networks, and mechanical strength. Repopulated cells in these decellularized whole-liver scaffolds are organized in a natural manner and perform a high level of biomimetic liver functions better than do conventional 2D culture systems [92]. Decellularized liver matrix is an ideal scaffold, but because of the complicated process, high cost, and concerns about the relevant differences between human and animal liver architecture and immunological reactions, the application of a decellularized liver matrix has some limitations [93].

For artificial scaffolds, we have more choices. The synthetic polymers are the basis of 3D scaffold culture, among which poly-lactic acid, poly-glycolic acid, and poly-caprolactone are the commonly used materials (Fig. 1). Especially, nanofibrous scaffolds formed by electrospinning are expected to be an ideal tool for tissue engineering because they are biocompatible scaffolds with topographic structures that can be fabricated to mimic the structures of natural ECM. Many studies showed that nanofibrous scaffolds are a good choice in regenerative medicine [94]. In addition, 3D bio-printing technology allows for the use of different materials to produce scaffolds with defined shapes and geometries. The generation of HLCs showed improved morphological organization, increased liver-specific gene expression, increased metabolic product secretion, and enhanced CYP induction in a 3D printed model. The application of bioprinting technology in tissue engineering allows for the development of a 3D biomimetic liver model that recapitulates the native liver module architecture and could be used for various applications such as early drug screening and disease modeling [95, 96].

However, the current methods for culturing organoids are usually costly and time-consuming. Scaffold-free approaches may overcome the problems. Some of the commonly used techniques are the hanging drop method, rotational culture or agitation, and use of low-adhesion plates to promote self-aggregation [97, 98]. To enable mass production of viable cell cultures, a bioreactor and a microwell array platform have been used for culturing organoids [81, 99]. As compared with the scaffold-based method, the scaffold-free model is simple and low-cost and implies no need to consider histocompatibility. Therefore, it is more suitable for large-scale drug screening.

#### Patient-derived organoids

The drug metabolic capacity of hepatocytes varies greatly among individuals. iDILI is often caused by poor metabolism or genetic disorders. iDILI is related to a variety of factors, so with animal tests and traditional models, predicting the hepatotoxicity of some drugs is difficult. One cannot conduct in vitro studies on PHHs from patients with iDILI; however, patient-derived organoids can be important tools for iDILI because iPSC-induced HLCs retain donor-specific CYP metabolism and drug responses [100]. Human organoids have been used to investigate infectious diseases, immune diseases, genetic diseases, and cancer. The use of organoids has led to the establishment of an in vitro personalized hepatic model system for disease modeling, drug discovery, and drug toxicity studies. For example, organoids from A1AT-deficient patients can be expanded in vitro and mimic in vivo pathology [101]. Ouchi et al. [102] successfully developed an organoid model of steatohepatitis. Using 11 different healthy and diseased pluripotent stem cell lines, the authors developed a reproducible method to derive multicellular human liver organoids composed of hepatocyte-, stellate-, and Kupffer-like cells that exhibited transcriptomic resemblance to the in vivo-derived tissues. Under free fatty acid treatment, these organoids successively recapitulated key features of steatohepatitis, including steatosis, inflammation, and fibrosis phenotypes. More importantly, organoids from patients with genetic dysfunction of lysosomal acid lipase phenocopied severe steatohepatitis and were successfully treated by suppression of farnesoid X receptor agonism-mediated reactive oxygen species. Furthermore, other disease models have been successfully established, such as rheumatoid arthritis [103], citrullinemia [104], and alcoholic liver injury models [105]. Thus, the patient-derived organoid platform is an effective tool for studying the mechanisms of disease and screening targeted drugs for human genetic disorders and allow for further progress in personalized treatment development.

#### Organ-on-a-chip

Organs-on-chips are microfluidic devices for culturing living cells in continuously perfused, micrometer-sized chambers that model the physiological functions of tissues and organs. The microfluidic system supplies a continuous flow of fresh medium and facilitates constant removal of metabolic waste, thus providing a consistent microenvironment to maintain cell viability and function over a long culture period. By manipulating the cell culture microenvironment with high precision, the efficiency of reprogramming human somatic cells into hiPSCs can be greatly improved [106, 107]. Wang et al. [108] established a liver organoid-on-a-chip system by using microengineering techniques, and the liver organoids exhibited dose- and time-dependent hepatotoxic responses after exposure to acetaminophen. Some experts believe that the microfluidic organoids for drug screening platforms may be cost-effective tools for the “fail early, fail cheaply” paradigm of drug development [109].

In vivo, organs and tissues do not exist in isolation but rather reside in a highly integrated and dynamically interactive environment in which they interact and support each other [110]. In addition to the liver-on-a-chip, a series of organs-on-chips, including the lungs [111], kidneys [112], intestines [113], and blood vessels [114], have been developed by use of microfluidic technology. Several laboratories have established multiorgan chips, such as liver–kidney coculture biochips and four-organ chips of the intestine, liver, skin, and kidney, which have shown a great advantage in evaluating pharmacokinetic and pharmacodynamic parameters [115–117]. For example, Schimek et al. [118] designed an integrated lung–liver organ chip. The authors found that aflatoxin B1, which has hepatotoxicity and carcinogenesis, impaired the function of lung tissues but had a protective effect when liver organoids were present. In contrast, in a multi-organ-on-a-chip system consisting of liver and cancer models, the anticancer prodrug capecitabine inhibited the proliferation of cancer cells after being metabolized by HepaRG cells [119]. Therefore, more complex drug metabolic reactions can be observed when several types of organoids are integrated into a single platform. The function of one organoid may influence the response of downstream organs, which is similar to how drugs are metabolized in vivo in that a drug may be metabolized by several organs [120]. Integrated multiorgan-on-chip systems will help further predict drug absorption, metabolism, and clearance in the body. However, with current technologies, replicating the exact size and function of each organ to accurately reflect the physiological interactions among them is challenging [121]. In addition, the human body is an integrated whole, and hormones, hemodynamics, and even biorhythms affect the metabolism of drugs in vivo. If the organ-on-chip system could consistently and accurately predict the pharmacology of drug candidates, organ-on-chip models might replace animal test models in the future [122].

### Hepatocyte-like cell models for in vivo hepatotoxicity testing

Drug metabolism differs in vitro and in vivo; therefore, preclinical evaluation of drug candidates in experimental animal models is an important step in drug development. However, owing to the differences between rodents and humans with respect to the metabolic and toxicological characteristics of drugs, accurately predicting the toxicity of drugs is often impossible [123]. To address this problem, chimeric mice with humanized livers were used for preclinical drug evaluation to replace traditional animal models [26]. Three types of chimeric mice with a humanized liver are frequently used for studies: urokinase-type plasminogen activator/severe combined immunodeficiency (uPA/SCID) mice, NOG mice expressing a thymidine kinase transgene (TK-NOG mice), and Fah^−/−^/Rag2^−/−^/Il-2rg^−/−^ (FRG) mice (humanized liver FRG mice) [124–126]. Immune deficiency and genetic modification in these mice allowed transplanted human liver cells to reproduce in the livers of these mice, resulting in chimeric mice with humanized livers that perform human drug metabolism and transformation functions [127].

Studies have found that the laboratory and histologic features of drug-induced liver toxicity in humanized mice mirrored those of humans [128–131]. For example, troglitazone is an antidiabetic drug that has been withdrawn from the market because of idiosyncratic severe liver injury. Its severe liver toxicity has never been induced in animal models until Kakuni et al. successfully detected it in chimeric mice with humanized liver [129]. Another study by Xu et al. [131] tested the dose-response of the drug fialuridine, a nucleoside analog for hepatitis B virus (HBV) infections, in humanized TK-NOG mice. Fialuridine did not display any toxicity in preclinical animal studies but was abruptly terminated in phase II clinical trials because seven of 15 clinical trial participants showed acute liver failure [132]. The authors found a dose-dependent liver toxicity in chimeric mice with a humanized liver as compared with non-humanized mice. Although currently most chimeric mice with humanized liver models used in hepatotoxicity testing (including the works of Kakuni et al. and Xu et al. mentioned above) were generated by transplanting PHHs [133–135], the use of stem cells to serve as hepatocyte sources for chimeric mice with a humanized liver is promising because stem cells are easily obtained and can be large-scale produced [136] (Fig. 1).

Stem cell-derived HLCs have been used to develop humanized liver HBV infection models in mice and evaluate anti-HBV drugs. For instance, Yuan et al. [137] developed an animal model with a human chimeric liver to study in vivo HBV infection by engrafting hiPSC-HLCs into Fah^−/−^Rag2^−/−^IL-2Rγc^−/−^SCID (FRGS) mice. As expected, the hHLC-FRGS mice reproduced HBV mimicking chronic HBV-caused viremia, and they were used to evaluate the effects of anti-HBV drugs. In the study, the combination of the well-demonstrated HBV entry inhibitor myrcludex B with the clinical drug entecavir efficiently blocked HBV spread in hHLC-FRGS mice. Similarly, the authors also used HepaRG cells to construct an HBV-infected humanized mouse model to evaluate anti-HBV drugs, including myrcludex B, cyclosporin A, vanitaracin A, irbesartan, and ritonavir and demonstrated that myrcludex B and cyclosporin A were more effective than the other three drugs in suppressing HBV replication [138].

Nevertheless, chimeric mice with humanized liver have some disadvantages. Generating chimeric mice with a humanized liver is costly and time-consuming [139]. And the efficiency of in vivo engraftment and expansion of immature HLC is still low. In the Yuan et al. study, FRGS mice implanted with HepaRG cells showed only about 10% liver chimerism, which was lower than that for PHHs [138]. However, in vivo administration of 5D5, an agonist c-Met receptor antibody, greatly promoted the expansion of hiPSC-HLCs in Fah-deficient mice, and the liver chimerism exceeded 40% in transplanted mice [140]. Nagamoto et al. [141] demonstrated that transplanted HLCs with overexpression of FNK (a hyperactive mutant gene from Bcl-xL) into uPA/SCID mice could enhance the repopulation efficiency of human liver chimeric mice. In addition, Ng et al. developed an inverted colloid crystal scaffold whose 3D mechanical properties could be engineered to reproduce the extracellular niche sensed by hepatic progenitors during human development. The model could help integrate, vascularize, and function the organoids following implantation into livers of immune-deficient mice [142].

## Conclusions

A large number of studies have shown that stem cell-derived hepatocytes have great potential in regenerative medicine, disease modeling, and drug screening. Only when the function of HLCs is consistent with that of PHHs can they accurately predict drug toxicity; hence, the differentiation of stem cells into fully functional hepatocytes remains a major challenge. On the one hand, small molecule compounds can replace the role of cytokines to improve the efficiency of differentiation [143]. On the other, researchers pay more attention to changing the microenvironment of cell culture to improve differentiation efficiency [144]. In recent years, with the development of 3D culture techniques, liver tissue engineering has been transformed from the classic monolayer cell culture to more advanced organotypic liver models that allow for more precise control of the microenvironment [145].

There are still many limitations to the use of 3D culture that need to be considered. First, the 3D model has not been able to replace the 2D culture model on a large scale [146]. Second, the results vary among laboratories [147]; therefore, the repeatability rate needs to be improved and the detection endpoints of cell differentiation and drug screening need to be unified. Third, according to the current protocols, generating organoids are time-consuming and costly [148]. To overcome these limitations, more technologies are needed, such as high-throughput microarray culture, 3D printing technology, and bionic scaffolds [149]. 3D culture combined with technology from materials science, bioengineering, and other fields will greatly improve the sensitivity and accuracy of drug screening.

In conclusion, the stem cell-based model provides an excellent platform for evaluating drug hepatotoxicity. In the future, combined with technologies such as gene-editing, omics, and single-cell sequencing, stem cell-derived HLC models will bring great benefits for drug toxicity and drug metabolism testing and also mechanisms of DILI and individualized medicine studies.

## Data Availability

All data are included in this published article.

## Abbreviations

DILI: Drug-induced liver injury
PHHs: Primary human hepatocytes
3D: Three-dimensional
2D: Two-dimensional
HBV: Hepatitis B virus
HLCs: Hepatocyte-like cells
hESCs: Human embryonic stem cells
hiPSCs: Human induced pluripotent stem cells
miRNAs: MicroRNAs
hMSCs: Human mesenchymal stem cells
hiHeps: Human-induced hepatocytes
DMSO: Dimethyl sulfoxide
CYP: Cytochrome P450
hECs: Human endothelial cells
ECM: Extracellular matrix
iDILI: Idiosyncratic drug-induced liver injury
FRG: Fah^−/−^Rag2^−/−^IL-2Rγc^−/−^
uPA/SCID: Urokinase-type plasminogen activator/severe combined immunodeficiency
